# Evidence That Head and Body Lice on Homeless Persons Have the Same Genotype

**DOI:** 10.1371/journal.pone.0045903

**Published:** 2012-09-26

**Authors:** Aurélie Veracx, Romain Rivet, Karen D. McCoy, Philippe Brouqui, Didier Raoult

**Affiliations:** 1 URMITE UMR 6236, CNRS-IRD, Faculté de Médecine, Université Aix-Marseille, Marseille, France; 2 MIVEGEC UMR 5290, CNRS-IRD-UM1-UM2, Centre IRD, Montpellier, France; Duke University Medical Center, United States of America

## Abstract

Human head lice and body lice are morphologically and biologically similar but have distinct ecologies. They were shown to have almost the same basic genetic content (one gene is absent in head lice), but differentially express certain genes, presumably responsible for the vector competence. They are now believed to be ecotypes of the same species (Pediculus humanus) and based on mitochondrial studies, body lice have been included with head lice in one of three clades of human head lice (Clade A). Here, we tested whether head and body lice collected from the same host belong to the same population by examining highly polymorphic intergenic spacers. This study was performed on lice collected from five homeless persons living in the same shelter in which Clade A lice are prevalent. Lice were individually genotyped at four spacer loci. The genetic identity and diversity of lice from head and body populations were compared for each homeless person. Population genetic structure was tested between lice from the two body regions and between the lice from different host individuals.

We found two pairs of head and body lice on the same homeless person with identical multi locus genotypes. No difference in genetic diversity was found between head and body louse populations and no evidence of significant structure between the louse populations was found, even after controlling for a possible effect of the host individual. More surprisingly, no structure was obvious between lice of different homeless persons.

We believe that the head and body lice collected from our five subjects belong to the same population and are shared between people living in the same shelter. These findings confirm that head and body lice are two ecotypes of the same species and show the importance of implementing measures to prevent lice transmission between homeless people in shelters.

## Introduction

Human head lice (*Pediculus humanus capitis*) and body lice (*Pediculus humanus humanus*) are obligate parasites; head lice live on the scalp and lay their eggs at the base of hair shafts, and body lice live on the body surface and lay their eggs on clothing [1]. Head and body lice are considered to be sub-species and are generally thought to colonize their host in an independent manner [2]. However, in circumstances involving people heavily infested with lice, such as in homeless populations, head and body lice are often found on the same person. This finding raises the question of whether the lice can migrate between the different body areas. Although numerous studies have attempted to elucidate this issue, the species status of these two types of lice is still debated [3].

Body lice pose a serious public health problem as they are vectors of the pathogens *Rickettsia prowazekii*, *Bartonella quintana* and *Borrelia recurrentis*, which are responsible for epidemic typhus, trench fever and relapsing fever, respectively [4], [5]. A comparison of the humoral and cellular immune responses of head and body lice following bacterial challenge showed reduced cellular (phagocytic) activity in body lice which may explain the higher level of vector competence that has been found in this subspecies [6]. The epidemiological role of head lice in the transmission of human pathogens has not yet been demonstrated, but several studies have reported the presence of *Bartonella quintana* in head lice [7]–[10]. It is therefore important to better understand the dynamics of human lice populations to minimize their propagation and the transmission of their associated pathogens in at-risk populations.

The first classifications of head and body lice were based on morphological characters. Some authors maintained that the morphological, behavioral and ecological differences between the two lice populations were not sufficient to recognize them as distinct species [1], [11]. Others, argued the reverse, that these differences required the recognition of these two groups as distinct taxonomic entities [12]–[15]. An analysis of primary endosymbionts indicated that these two types of lice are conspecific [16], but louse isoenzymes suggested that genetic differentiation may exist between the two forms [17]. After these phenotypic studies, numerous DNA-based molecular studies were performed, and again presented conflicting conclusions [3], [18], [19]. Currently, three deeply divergent clades (or phylotypes) of human lice with different geographic distributions are recognized: clades A, B and C. Phylotypes B and C contain only head lice, but phylotype A includes both head and body lice [20], [21]. Clade A lice have been further subdivided into subclusters of non-Sub-Saharan African lice (called A1) and Sub-Saharan African lice (called A2), as reported by two independent studies. The first study was based on the 18S rRNA gene sequence [22] and reported the divergence of head and body lice as being a recent event that occurred independently in each geographical group. The second study was based on the PM2 spacer [23] and could not show head and body louse divergence within each of the two clusters. Head and body lice were also shown to be genetically indistinguishable in a worldwide study based on four intergenic spacers [24] and in a very recent study based on the louse transcriptome [25]. Finally, based on a Bayesian coalescent model, ancestral migration events between head and body lice were shown to happen in both directions [26].

As multispacer typing was shown to be useful in addressing population-level questions [24], we used this genotyping method to determine if homeless people were infested by head and body lice of the same population. We examined the genetic population structure between lice from two body regions of five human subjects. However, one of the critical problems associated with this experimental design is that lice can migrate temporarily from one site to the other (with or without reproduction), making it difficult to determine their true origin (head or body). Consequently, to avoid any possible confusion regarding the origin of the tested lice, we collected eggs from the hair and clothing of homeless people from one shelter in Marseille, France. After hatching these eggs in the lab, we genotyped the first instar larvae and tested the genetic population structure of the lice from the two body areas.

## Methods

### Ethics statement

In Marseille, there are an estimated 1500 homeless people, and 600 of them sleep in one of two available shelters (A and B) [27]. Because these individuals live in poor sanitary conditions, homeless persons are exposed to a number of health problems and belong to the social class with the most limited access to healthcare. To implement appropriate preventive and curative interventions, a snapshot investigation of the two shelters of Marseille has been performed each year since 2000 by a multidisciplinary team [28], [29]. The study protocol was reviewed and approved by the Institutional Review Board and Ethics Committee of Marseille No. 10.005 as it is in accordance with the French Bioethics law N° 2004-800 60 (06/08/2004). The study reported here was made based on samples collected in 2010. Homeless persons were informed of the purpose of the intervention and were asked if they would agree to participate by reading and signing an informed consent form . The document was divided into two parts: one for the patient with all information about the study and the other part including patient signature was kept by the investigators. The homeless persons were then interviewed and given a physical examination by a medical doctor. A nurse collected blood and other microbiological samples. One of the researchers (AV) was assigned to this team to meet the homeless and to collect head and body lice. When an individual had a body louse infestation, we provided clean clothes and kept the lice-infested undergarments and T-shirts in a sealed container to later harvest the eggs. In the cases of head louse infestations, the hair was cut and used to harvest the eggs. The infested homeless person was then invited to take a shower and was offered treatment with ivermectin [30]. The investigations consisted in a clinical exam that was offered to any homeless who presented even if he would not agree to participate to our study. Every homeless including participating and non-participating persons were offered the same services and a prescription was given if needed. Moreover, depending on the results of the samples analysis, the patient was taken in charge in the hospital if needed. All homeless in France are eligible for a social security cover (free healthcare for people on low incomes), this permit us to include all potential participants.

### Eggs incubation before hatching

In the laboratory, the infested clothes were cut to separate the collar from the rest of the clothes. Eggs situated on ball caps (Figure 1A), collars (Figure 1B) or beards were not included in the analysis to avoid using lice located on the “borders” between head and body lice. The fabric and hair that contained eggs were put in labeled and separated boxes with holes, and grouped by the homeless person that they were isolated from. All of the eggswere incubated at 29 degrees Celsius with 70 to 80 percent relative humidity until hatching. Each day for 8 days, the newly hatched larvae were collected and stored at −20°C until further processing. Figure 2 shows a head louse (Figure 2A) and a body louse (Figure 2B) with their respective nits (empty egg shells) one day after hatching in the laboratory.

**Figure 1:** Lice eggs attached to a homeless cap (A) and a homeless collar (B).

**Figure 2:** Picture of a head louse (A) and a body louse (B) and their respective nits.

### Genotyping

Total genomic DNA extraction, PCR and sequencing of the intergenic spacers S2, S5, PM1 and PM2 were performed as described previously [23]. As lice are diploid, cloning was necessary to identify the different allelic sequences; therefore, PCR products were cloned using a previously described protocol [23]. The resulting sequences were aligned with genotypes published in GenBank [23], [24] for identification. When less than 100% homology was obtained, the new genotype was recorded, a new number was assigned to it and it was published in GenBank (JX041640–JX041654). This was done according to a new set up of GenBank submissions providing the gene names that this is the intergenic spacer between: PHUM005704-PHUM006210 for intergenic spacer 2 , PHUM007351-PHUM002191 for intergenic spacer 5, PHUM007934-PHUM003340 for intergenic spacer PM1 and PHUM002215-PHUM002223 for intergenic spacer PM2

We also used high-throughput 454 sequencing of the amplicons using tagged libraries. Libraries were created by PCR using the same protocol as above and the same specific primers with the addition of the 454 adaptor and a Multiplex Identifier sequence (MID). The same 8 nucleotide barcode was used for all primer pairs (spacer S2, S5, and PM2). A total of 13 barcodes were designed using *Barcrawl* software [31]. We excluded barcodes with the same 5′ base as 3′ end of the upstream 454 adaptor, and we added a guanine to the 3′ end of the barcode to avoid the presence of the same 3′ barcode base at the 5′ end of the downstream primer. Barcodes that were converted to other barcodes by deletion were excluded. The numbers of 454 GS-FLX nucleotide flows to sequence the barcodes were as low as possible and were used between 5 and 9 flows (Supplementary Tables 1 and 2). The preparation of the 163 libraries was performed, as described in the Amplicon Library Preparation Method Manual from Roche. Additionally, 8 pools of 20 to 21 libraries were created to perform the clonal amplification, as described in the emPCR Method Manual from the Lib-A SV GS FLX Titanium Series from Roche. We worked with two Small Volume Emulsions of capture beads A and two Small Volume Emulsions of capture beads B per pool of libraries at a ratio of 1.8 copies of library per bead. The sequencing was performed in accordance with Roche using a GS FLX Titanium sequencing Kit XLR70 and the PicoTiter plate that was divided into 8 medium-sized regions.

**Table 1:** Diversity estimates for each locus and population of lice from the bodies and heads of the sampled homeless persons.

Locus	Diversity	Host S		Host 33		Host F		Host M		Host D	
	estimate	Body	Head	Body	Head	Body	Head	Body	Head	Body	Head
		(n = 17)	(n = 2)	(n = 6)	(n = 9)	(n = 5)	(n = 4)	(n = 5)	(n = 3)	(n = 5)	(n = 9)
**S2**	***h***	0.836	0.500	0.833	0.764	0.650	0.708	0.875	0.667	0.667	0.804
	**π**	0.025	0.011	0.029	0.033	0.029	0.012	0.037	0.009	0.008	0.030
**S5**	***h***	0.669	0.000	0.667	0.743	0.375	0.833	0.675	1.000	0.667	0.518
	**π**	0.024	0.000	0.024	0.026	0.006	0.024	0.024	0.033	0.028	0.009
**PM2**	***h***	0.836	1.000	1.000	0.722	0.700	1.000	1.000	0.833	0.875	0.736
	**π**	0.011	0.010	0.009	0.005	0.006	0.007	0.012	0.007	0.004	0.005

Gene diversity (h) and nucleotide diversity (π) are based on Nei's (1987) estimates.

n refers to the number of lice genotyped for each locus.

**Table 2:** Summary of Hardy-Weinberg tests when louse populations are defined at the level of the body location of each homeless person (head or body), or when combined across body locations for each homeless person.

Dataset	Locus	n	Fis (SE)	P-value
***Body location***	**S2**	10	0.2210 (0.1688)	0.1809
	**S5**	9	0.5843 (0.1328)	0.0003
	**PM2**	10	0.6782 (0.0862)	<0.0001
	**Overall**	29	0.4914 (0.0835)	<0.0001
***Homeless person***	**S2**	5	0.3306 (0.0609)	0.0032
	**S5**	5	0.5891 (0.1047)	<0.0001
	**PM2**	5	0.6222 (0.1138)	<0.0001
	**Overall**	15	0.5140 (0.0620)	<0.0001

P-values represent the combined value across populations (Fisher's procedure).

n refers to the number of combined values.

Fis (± standard error) refers the average unweighted value across populations and measures the deviation from panximia.

For each region, barcodes were associated with only one DNA sample. We used *mothur* software [32] to trim the sequences and identify the barcodes using the following parameters: *minlength = 100, bdiffs = 1, qwindowsize = 50, qwindowaverage = 25* (Supplementary Table 3). The trimmed sequences were mapped to the 3 reference genes using the program CLC Genomics Workbench. A probabilistic variant table was created for each mapped gene and every SNP (small nucleotide polymorphisms) and DIP (deletion and insertion polymorphisms) were verified and associated to extract the two alleles.

**Table 3:** Analysis of molecular variance (AMOVA) of louse populations for each spacer locus.

Locus	Level	df	% variation	Fixation index	P-value
**S2**	**Among homeless persons**	4	0.31	Fct = 0.0031	0.57283
	**Between body locations (homeless)**	5	9.25	Fsc = 0.093	0.06647
	**Within body locations**	114	**90.45**	**F**st** = 0.096**	**0.00782**
**S5**	**Among homeless persons**	4	10.84	Fct = 0.11	0.14374
	**Between body locations (homeless)**	5	11.30	Fsc = 0.13	0.19129
	**Within body locations**	116	**77.86**	**F**st** = 0.22**	**0.00759**
**PM2**	**Among homeless persons**	4	5.11	Fct = 0.051	0.12401
	**Between body locations (homeless)**	5	4.48	Fsc = 0.047	0.58660
	**Within body locations**	116	90.41	Fst = 0.096	0.08566

% variation indicates the amount of overall variation in the data explained at a given level of organization.

The fixation indices refer to the amount of genetic structure attributed to each level.

It should be noted that at the Within body locations level, the % variation refers the amount of variation found within populations,

whereas Fst measures the structure among populations.

% variation indicates the amount of overall variation in the data explained at a given level of organization.

The 454 sequencing results were blasted against the results obtained from the PCR and cloning method. Differences in numbers of A or T in homopolymers were not taken into account.

### Population genetic structure

The genotypic data were analyzed using tests based on both the allelic identity and the allele sequence. For the tests based on allelic identity, each unique sequence was assigned an allele number and the genetic distance among the sequences was considered equal. Using these data, we first tested to see if Hardy-Weinberg proportions (HW) were found within the populations. To determine the correct level of a population, we tested for HW by using two different combinations of the sampled lice. First, we broke the lice into the smallest possible biological unit by grouping all lice from a given body area on a given homeless person (body location data, n = 10 populations). Next, we considered all lice from the same homeless person as representing as single population, regardless of whether the lice were found on the head or body (homeless person data, n = 5 populations). If there was significant isolation between head and body lice, we expected to find higher deviations from HW in the latter case due to a Wahlund effect [33]. Deviations from the expected HW proportions for each population and locus were measured by Weir and Cockerham's estimator of Wright's Fis index and tested for significance using exact probability tests implemented in the software GENEPOP v4.1. Exact p-values were calculated using the Markov chain method, and tests across body locations, individuals and loci were combined using Fisher's procedure [34].

Gene diversity and nucleotide diversity was estimated for each locus and population using the body location dataset and the software *F-STAT v 2.9.3* [35] and Arlequin v.3.5.1.3 [36], respectively. Differences in diversity among head and body lice were tested using paired t-tests for each locus. Tests across loci were combined using Fisher's procedure [34].

We used the sequence-based genotypic data to carry out an Analysis of Molecular Variance (AMOVA) that considers the allelic content of the genotypes and their frequencies to measure the population structure at different hierarchical levels of organization (i.e., within populations, among populations within groups, among groups) [37]. This analysis was carried out using the software *Arlequin v.3.5.1.2* [36] and tests for the significance of the covariance components associated with each organizational level were performed using a non-parametric permutation procedure (20,000 permutations of the data where the type of permutation depends on the organizational level). This analysis also provided fixation index estimates for each level, ie, a measure of population structure [38].

## Results

### Collections

During our investigations, not all homeless people were willing to cooperate, either because the rooms of the shelters were cold and not comfortable enough to allow them to change clothing or because they preferred to have their meal and go directly to bed. Additionally, because of the regular head shaving of homeless diagnosed with head lice that had been previously offered, we had difficulty finding head lice on many of the individuals. The presence of head lice was most frequently noted on hair near the neck or above and behind the ears. For body lice, we noted that eggs and even motile forms were found much more often near seams, particularly in the armpit.

During our investigations, we met 210 homeless people. Among them, 29 subjects had lice with 2 who had only head lice, 14 had only body lice and 13 had both. In addition to the head lice, we collected 163 body eggs (with 44 attached on the collar) and 727 mobile forms (larvae or adults). The head lice that we collected included 116 head eggs (with 10 attached to the beard) and 340 mobile forms. However, genotyping was only performed on the first instar larvae that were hatched from the eggs collected from homeless persons that had both head and body eggs. These criteria left us with 38 body lice larvae and 27 head lice larvae from 5 homeless people that were all sleeping at shelter A. Interestingly, we never found body lice eggs without larvae or adult body lice on the same body. In contrast, some homeless people had head lice eggs without larvae or adults found in hair (among our 5 studied homeless subjects, this is the case of homeless person S).

### Genotyping

The PM1 spacer region was monomorphic (genotype 13) for all of the genotyped lice and was therefore not included in the analyses. Many of the collected lice were heterozygous as multiple sequences were overlaid in the chromatograms. For these individuals, cloning was needed to assess the genotypes. This was the case for almost all of the S2 sequences, many of the PM2 sequences and some of the S5 sequences. To ensure that all genotypes had been correctly assessed, the results obtained from the PCR and cloning method were compared with the results obtained from the high-throughput 454 sequencing of the same samples. In general, our results were congruent. However, it happened very often that the number of Ts or As found in homopolymers varied. Indeed, the polymerase can easily make mistakes at these positions, resulting in differences between the two sequencing methods and even between different clones or reads generated by the same sequencing method. Differences in homopolymer length were therefore not taken into consideration in the analyses. Moreover, the cloning method is long and fastidious when sequencing diploid organisms. The 454 sequencing method offers many advantages, including the production of hundreds of clones in one step. However, in some cases the reads obtained were not long enough to cover the studied region, so some adjustments to the protocol or to the chosen primers might prove useful. Overall, the sequencing run produced 285,002 reads with an average length of 484.5 nt and a median length of 507 nt. The total number of bases sequenced was 138,103,874, and the average quality score was 26.98.

As shown in figure 3, we observed that the majority of genotypes, including the most common genotypes, were shared between head and body lice (in green). The most prevalent alleles in head and body lice were the same. For the PM2 spacer region, alleles 1, 38 and 33 were present in the majority of lice. In spacer S5, the more frequent alleles were 42 and 12. Finally, in spacer S2, the most frequent alleles were 48 and 68 (Figure 3). The raw data are provided in Supplementary Table 4. The concatenated genotypes of the S2, S5 and PM2 spacers that occurred at least twice in our sample are presented in Figure 4. We found two pairs of head and body lice on the same patient (homeless person 33) that had a unique multi-locus genotype, indicated with green arrows in Figure 4 (genotype 68, 42, 33 and genotype 68, 42, 48). This suggests that related individuals can be found on both regions of the body.

**Figure 3:** Proportion of each allele among the head and body lice. The names (ID numbers) of the alleles are mentioned followed by the letter H for head lice and B for body lice. The alleles found in both the head and body lice are shown in green. The blue alleles were found only in the head lice, and the yellow alleles were found only in the body lice.

**Figure 4:** Repartition of head and body lice haplotypes found at least twice in our samples. The haplotypes are concatenated alleles of the S2, S5 and PM2 spacers. A single color was assigned to each unique haplotype. Each block represents one louse, but may be separated into several colored units if the alleles at the three spacers could be combined to generate multiple haplotype possibilities. The green arrows indicate identical head and body lice haplotypes collected from the same homeless person.

### Genotypic data analyses

Genetic diversity and nucleotide diversity were similar among the head and body lice populations sampled from the homeless individuals (Table 1; Fisher's combined test Chi^2^ *_h_* = 2.323, df = 6, *P* = 0.888; Chi^2^ *_π_* = 4.616, df = 6, *P* = 0.594). HW proportions were not found within lice populations. Indeed, the fixation index (Fis value) was positive (indicating a deficit in heterozygotes), and significant in almost all cases regardless of the spatial organization of the data (Table 2). Only the estimate for locus S2 was non-significant when populations were considered at the level of the body location, but this change is most likely caused by the high standard error of this estimate associated with the reduced population sizes of lice populations when divided into two groups for each homeless person. Indeed, restricting a louse population to only those lice found on the respective head or body zones of a given homeless person did not significantly reduce the overall heterozygote deficits present in the dataset (Table 2) and suggests that deficits at the homeless person level are not due to a Wahlund effect, i.e., an artifact of mixing different isolated populations.

AMOVA analyses revealed no significant population structure between head and body lice after controlling for the sampled person at any of the three loci tested (Table 3). Indeed, the fixation index at this level of population organization was low (Fsc) and non-significant. Furthermore, no structure was evident among lice of different homeless persons (Fct). However, some population structure was evident among all populations (Table 3, Fst), but detailed pairwize comparisons could not reveal any interpretable pattern to this structure (data not shown). This structure may therefore be due different colonization histories and drift among some of the head and body populations.

## Discussion

In people infested with both head and body lice, the original ecosystem of the lice can be dubious. Indeed, we found numerous eggs on collars, beards and ball caps that could have been from either the head or body (Figure 1). The method used to sample the two types of lice is therefore critical. For this reason, eggs collected from hair (head lice) and eggs collected from clothes (body lice) were kept separate and incubated until hatching, and molecular analyses were performed on the newly hatched larvae. All precautions to avoid DNA contamination were taken, and negative controls were used at each step of the study. Moreover, the use of two sequencing approaches strengthened our results because both techniques were concordant. Based on this data, and despite the elimination of individual lice in the potential overlap zones, our results strongly suggest a genetic mixing of lice from head and body populations.

After genotyping lice, the genetic diversity and the nucleotide diversity was calculated for each spacer and used to compare head and body lice populations. This was not calculated for the spacer PM1 because it was monomorphic in the tested populations. The spacers S2, S5 and PM2 showed high heterogeneity in both the head and body lice (Table 1). However, these two groups of lice did not differ significantly in gene diversity or nucleotide diversity at the studied loci. This contrasts with a previous study that reported a higher nucleotide diversity in head lice compared to body lice [39]. This may be caused by a sampling bias as this previous study was based on 40 lice collected from across 12 different countries. We also found two pairs of head and body lice with identical genotypes collected from the same homeless person (homeless 33) (Figure 4) suggesting that related individuals move between body areas on the host.

Strong heterozygote deficits were present in all populations, regardless of how a population was defined (all lice from a given homeless person, or only those lice from the respective head or body populations). This result is not surprising given that transmission ratio distortion, that is, a non-Mendelian inheritance pattern of alleles, is known to occur in *P. humanus* populations and may have caused the HW disequilibria found in this study [40]. However, regardless of the presence of this distorter, the deviation from HW equilibrium proportions at the level of homeless person was not reduced by dividing lice into the smallest possible population unit, that of the body zone within a host individual. Although it is possible to have a Wahlund effect due to mixing of different louse families within each body zone, no Wahlund effect seems to be related to mixing lice from head and body populations on single host. These results are further supported by those of the AMOVA analyses which showed little genetic variation attributable to between host and body lice populations and no significant structure between these populations.

These results validate previous assumptions that the clade A lice may evolve and colonize both the hair and clothing niches [24], [25]. First, our results suggest that the lice collected from our five subjects belong to a single population and, thus, that lice are shared between people living in the same shelter. They further indicate that head and body lice likely move frequently from one part of the body to the other. These results support recent data comparing the transcriptional profiles of head and body lice [25]. Fourteen putative differentially transcribed genes were identified between head and body lice that could explain phenotypic differences [25]. The presence of two clades of lice living on some host individuals may help explain previous reports of independent head and body lice population [9], [19]. Indeed, a study on doubly infested persons in Ethiopia showed that all of the head lice were black and of clade C and all of the body lice were gray and of clade A [9]. Moreover, the only other study that reported independent head and body lice populations on individuals infested by the two forms was undertaken in Nepal where both Clade A and C lice are prevalent [19]. In the case of the clade A lice from our study, it seems that migration occurs between the two body zones and that it may increase in case of massive infestations. However, here we consider only lice that hatched from collected eggs. It remains to be shown whether these individuals could durably establish in the ecological niche where they were found. From our data, we can also not say whether migration is bidirectional between body zones (from both head to body and body to head) or whether one zone acts as a source for the other. However, a previous study showed that a single gene of an unknown function seems to be lost in all head lice [25]. This finding suggests that head lice may originate from body lice rather than the reverse. More complete phylogeographic studies are called for to test this hypothesis.

Our failure to find population structure among homeless persons living in the same shelter may indicate that louse transmission frequently occurs in shelters. Prevention measures should therefore focus on avoiding the sharing of items such as mattresses, blankets and other personal belongings through which lice transmission is likely to occur from one homeless person to another.

## Supporting Information

Table S1 **Primer sequences.**
(XLS)

Table S2 **Barcode sequences.**
(XLS)

Table S3 **Recovery statistics after Mothur processing.**
(XLS)

Table S4 **Results of the Multi-Spacer-Typing of homeless lice.**
(XLS)
